# Uses of Different Machine Learning Algorithms for Diagnosis of Dental Caries

**DOI:** 10.1155/2022/5032435

**Published:** 2022-03-31

**Authors:** Sarena Talpur, Fahad Azim, Munaf Rashid, Sidra Abid Syed, Baby Alisha Talpur, Saad Jawaid Khan

**Affiliations:** ^1^Department of Biomedical Engineering, Ziauddin University, Karachi, Pakistan; ^2^Department of Electrical Engineering, Ziauddin University, Karachi, Pakistan; ^3^Department of Software Engineering, Ziauddin University, Karachi, Pakistan; ^4^Liaquat University of Medical and Health Sciences, Jamshoro, Pakistan

## Abstract

**Background:**

Dental caries is one of the major oral health problems and is increasing rapidly among people of every age (children, men, and women). Deep learning, a field of Artificial Intelligence (AI), is a growing field nowadays and is commonly used in dentistry. AI is a reliable platform to make dental care better, smoother, and time-saving for professionals. AI helps the dentistry professionals to fulfil demands of patients and to ensure quality treatment and better oral health care. AI can also help in predicting failures of clinical cases and gives reliable solutions. In this way, it helps in reducing morbidity ratio and increasing quality treatment of dental problem in population.

**Objectives:**

The main objective of this study is to conduct a systematic review of studies concerning the association between dental caries and machine learning. The objective of this study is to design according to the PICO criteria.

**Materials and Methods:**

A systematic search for randomized trials was conducted under the guidelines of PRISMA (Preferred Reporting Items for Systematic Reviews and Meta-Analyses). In this study, e-search was conducted from four databases including PubMed, IEEE Xplore, Science Direct, and Google Scholar, and it involved studies from year 2008 to 2022.

**Result:**

This study fetched a total of 133 articles, from which twelve are selected for this systematic review. We analyzed different types of machine learning algorithms from which deep learning is widely used with dental caries images dataset. Neural Network Backpropagation algorithm, one of the deep learning algorithms, gives a maximum accuracy of 99%.

**Conclusion:**

In this systematic review, we concluded how deep learning has been applied to the images of teeth to diagnose the detection of dental caries with its three types (proximal, occlusal, and root caries). Considering our findings, further well-designed studies are needed to demonstrate the diagnosis of further types of dental caries that are based on progression (chronic, acute, and arrested), which tells us about the severity of caries, virginity of lesion, and extent of caries. Apart from dental caries, AI in the future will emerge as supreme technology to detect other diseases of oral region combinedly and comprehensively because AI will easily analyze big datasets that contain multiple records.

## 1. Introduction

Dental caries is known as tooth decay, and it is a disease of damaging the teeth that is caused by bacteria in the mouth making lactic acids that directly affects tooth surface layer known as enamel layer. Slowly and gradually, this can lead to a small hole or cavity in teeth; if this is not treated, it will cause pain, infection, and eventually loss of tooth [1–3].

Dental caries is a major problem of oral health in most developing and underdeveloped countries. According to World Dental Federation (FDI), oral diseases affect about 3.9 billon people; among them 60–90% affect school children. A massive majority of adults, nearly 100%, have tooth decay that often leads to pain and discomfort. Untreated dental caries impact almost 44% of world population [4] and will make it the most prevalent disease in all 195 countries of the world. Centre of Disease Control and Prevention (CDC) estimates in USA that the morbidity rate among persons aged 6–19 years is 16.9%, whereas in adults aged from 22 to 24 years, it is increased by 31.6% [3].

Some of the earliest studies worked on conventional methods or systems for the diagnosis of dental caries by using visible light transillumination method [5], tuned aperture computed tomography [6, 7], international caries detection and assessment system [8], and quantitative light-induced fluorescence [9]. Other studies developed a system to modify the dental panoramic radiology by using some image processing technique for the diagnosis of dental caries. Some studies are using edge detection task by using Gaussian filter [10], conventional digital imaging [11, 12], near-infrared imaging [13], and semisupervised fuzzy clustering methods [14]. Although during the past few decades the prevalence of dental caries has fallen dramatically, its detection still remains a big challenging task for many experts.

Artificial intelligence is sometimes called machine intelligence, and it is revealed by a machine undistinguished by human's and animal's intelligence. It has a broad spectrum of introducing advanced technologies that make daily life easy. The evaluation of machine learning provides reliable information and helps in improving decision-making processes in medical field [15]. The major goal of AI is to permit automated learning without the involvement of human judgement. The model of AI can predict future outcomes with the help of initial data. The model of AI is illustrated in Figure 1.

Like other fields, AI also emerged in the field of dentistry. It can perform simple and complex tasks in dental clinic with greater precision, accuracy, sensitivity, and, most importantly, lesser time [16]. For example, AI can automatically detect caries, bony lesions, and maxillofacial abnormalities from dental radiographs without the involvement of any dentist in lesser time and with more accurate results. So, dentists can recognize diseases comparatively easily.

Computer-based diagnosis is increasing momentum because of its capabilities in diagnosis of lesion and caries, which may not be seen by naked human eye. The various techniques that are applied to dentistry especially for detection of caries include adaptive neural network architecture [17], deep learning [18], an artificial multilayer perceptron neural network [19], convolutional neural network [20], backpropagation neural network [21], and *k*-means clustering [5]. By using these techniques, a big, challenging task has been observed to be vanished. So, in this systematic review, we will discuss various artificial techniques that are used to detect dental caries.

The objective of this paper is to conduct a review of studies concerning the association between dental caries and machine learning according to PICO criteria (population, intervention, comparison, outcomes), where the following hold:

1. Population (P): Dental X-ray images of human beings.
2. Intervention (I): Analysis of the different algorithms of machine learning used to detect dental caries.
3. Comparison (C): Different algorithms of machine learning to predict the caries.
4. Outcomes (O): Accuracy of algorithms.

## 2. Methodology

This research is fully investigated under the guidelines of PRISMA that lists items for systematic review and meta-analysis.

### 2.1. Source

An e-search was conducted via PubMed, IEEE Xplore, Science Direct, and Google scholar databases. The key terms that were used for electronic search were “Dental Caries” and “Machine Learning” with AND operator. The e-search was limited to the studies that were published between the years 2008 and 2022 and included only human studies. We also restricted our search to patent and citation.

### 2.2. Study Selection

This systematic review mainly focused on original papers that applied different algorithms of machine learning to predict any type of dental caries.

### 2.3. Inclusion Criteria

The following set of inclusion criteria was made to collect relevant information from various researches to fulfil the objectives of this review paper.

1. Research papers must be written in English language.
2. The studies must be limited to human dental health.
3. All papers must be published between the years 2008 and 2022.
4. Research papers specify the size of datasets in their studies.
5. Research paper specifies clear explanation for the detection of caries through machine learning.
6. Research papers provide information of various machine learning parameters like accuracy and classifier techniques in diagnosis of dental caries.
7. Can be a conference paper of IEEE.

### 2.4. Exclusion Criteria

The following exclusion criteria were used to eliminate irrelevant information sources.

1. Non-English papers.
2. Research papers that included machine learning for dental X-ray image segmentation and to identify oral health.
3. Studies that related dental caries detection with any image processing tool.
4. Those studies that specified other dental diseases like oral cancer and sensitivity of teeth.
5. Conventional methods like ICDAS (International Caries Detection and Assessment System) detection of dental caries through visualization of X-ray radiographs.
6. Reviews papers, systematic reviews, meta-analysis, thesis and dissertations, letters, editorials, abstracts, unpublished studies, case reports, small case series, and cross-sectional studies.

### 2.5. Risk of Bias Criteria: Quality Assessment of the Studies

The quality assessment of the studies was performed on the basis of the following keys items.

1. Inclusion criteria
2. Exclusion criteria
3. Feature extraction criteria
4. Description of the diagnosis of dental caries
5. Radiographic examination for dental caries diagnosis
6. Machine learning algorithm description
7. Samples of dataset >149
8. Description of testing and training evaluation:
9. Training = equal to or less than 70%
10. Testing = equal to or greater than 30%
11. Statistics and evaluation

### 2.6. Data Extraction

The selected research papers presented important information involving techniques of machine learning to predict caries in human teeth along with various parameters related to it. The following data was found to be significant on the literature evaluation and therefore these parameters were scrutinized for each research paper: author names, year of publication, country, size of datasets of X-dental images, algorithm, classifier, objectives, language, and accuracy.

Other factors like feature extraction from the dataset of X-ray dental images can also reduce data repetitiveness of analysis of dataset that directly fascinates machine learning, informs various features combinations, and results in increasing speed of learning and necessary steps in the process of machine leaning. However, due to the unavailability of complete data in the searched research papers, theses parameters could not be included for analysis.

## 3. Results

One hundred thirty-three articles were fetched from electronic search: 70 from Google Scholar, 8 from IEEE Xplore, 20 from PubMed, and 35 from Science Direct. Exclusion of articles was based on five phases.

The first phase consisted of removing the duplication of articles where only eighty-eight articles were taken. After removing duplicated articles, the second phase was the evaluation of title screening; only forty-five articles remained. However, the third phase was the assessment of abstract; twenty-two articles were selected from it. The fourth phase was the eligibility of full-text articles; only eighteen articles were selected. The fifth phase (selection of articles that were included into this systematic review paper); six out of eighteen articles were excluded due to missing/irrelevant data. Only twelve articles were selected.

### 3.1. Table for Risk of Bias Assessment

Risk of bias assessment is summarized in Table 1.

### 3.2. PRISMA Flow Diagram for Present Systematic Review

PRISMA flow diagram for present systematic review is shown in Figure 2.

### 3.3. Characteristic Table for the Selected Studies

Characteristic Table for the selected studies is shown in Table 2.

In all selected studies, deep learning with algorithms CNN and ANN was used as a major component of network to detect dental caries. Other types of network used in these studies were hidden layer propagation, Support Vector Machine, Random Forest, Logistic Regression, feedforward propagation and feedback propagation, CNN- and ANN-based research. Deep learning-based papers have appeared in the field of dentistry to detect and diagnose the dental caries since 2008 and more papers using deep learning specially CNN have been published.

The size of dataset that was used for training and testing data also increased from 80 to 9630 and from 80 to 2380, respectively, up to 2019, but in 2020, there is no clearly maintained description for training and testing data. After the year 2020, the ratio of using training and testing data also decreased by 2387 and 603, respectively, in the years 2021 and 2022 (see Figures 3 and 4). This variation in the data size is simply based on selection of dataset in respective studies.

Although these studies contribute more to dentistry, these were restricted only to the diagnosis of three types of caries: proximal, root, and occlusal. A few papers only detect the presence of caries in human teeth whereas one among these studies diagnosed the existence of bacteria *Streptococcus mutans*, indicating the initial stage of caries.

In addition to this, different types of imaging modalities have been studied; coherent with these studies, the only reason was to extract feature to diagnose dental caries by using 2D and 3D radiographs.

## 4. Discussion

Computer-Assisted Diagnosis (CAD) has been used in medical field to obtain suggestions, but the designing and tuning of these old techniques of CAD tend to be very difficult. Nowadays, artificial intelligence (AI) techniques have been integrated into these computer-based diagnoses in order to get accurate and fine results for different branches of medical field. The qualitative and quantitative approaches of AI in dentistry increase day by day. Some areas need to be emphasized to expand the continuous advancements of artificial intelligence research in detecting dental caries.

The studies that were selected for this systematic review were the ones that satisfied at least 70% of quality assessment criteria. Out of various studies that correlate AI and dental caries, only twelve were selected for the analysis.

It has been noticed that various different factors can influence the contrast between selected and nonselected studies, for example, conventional methods (isophote concept, ICDAS, tuned aperture computed tomography, and image processing) with artificial intelligence techniques. Also, what influences is the comparison among selected researches. For example, sample size ranges from 45 to 3000 between individual studies. Accuracy and type of dental caries also differed from one study to another.

Previously, review article demonstrated the causes of dental caries, biomarker for dental caries, or relation with other factors, like obesity and nutritional features, and provided overall overview of deep learning in dentistry field [15, 22, 23]. Our investigation for this review emphasizes only on detection of dental caries by different algorithms used in artificial intelligence. Unlike other review articles that are general to dentistry (means involved application of machine learning in all the subfields of dentistry), this review paper restricted studies only to dental caries. In this way, we analyzed performance with accurate results and efficiency in the diagnosis of tooth caries rather than approaching for the automatic teeth segmentation, dental radiographs segmentation process, and detection of caries all in one review article.

The data for this review was investigated in order to analyze different algorithms of machine learning used to detect caries. Table 1 shows the characteristic for this systematic review and includes only twelve studies from time period 2008–2022.

We observe that all the selected studies support deep learning or deep neural network for caries detection, a member of a broader family of machine learning, including backpropagation [19, 24], fully convolutional neural network (CNN) [25, 26], convolutional neural network [18, 27], mask CNN [28], support vector machine [29, 30], and artificial neural network (ANN) [31].

Patil et al. [17] evaluated the best algorithm used for the diagnosis of tooth caries, and they determined the best algorithm by showing the relationship among support vector machine (SVM), *k*-nearest neighbor (KNN), Naïve Bayes (NB), and adaptive dragonfly algorithm (ADA-NN). They took a sample size of 120 dental images and performed three tests on 40 dental images each. Every time ADA-neural network showed the best performance in comparison to other mentioned algorithms (resp. 5.5%, 11.76, and 6.5% better than others).

Javed et al. [31] used feedforward backpropagation with a sample size of 45 molar teeth images to predict post-*Streptococcus mutans* as it is a primary initiator and one of the most common microorganisms associated with dental caries. The study used another method of deep learning and justified their studies by claiming 99% of accuracy in predicting the presence of bacteria in premolar teeth.

Two researches from the selected studies, by Devito et al. [19] and Geetha et al. [21], used backpropagation algorithm of deep learning to predict dental caries. Devito et al. [19] expanded their study in predicting proximal type of dental caries from X-dental radiographs with an accuracy of 88.4%.

Similarly, another study by Casalegno et al. [18] used a sample size of 217 X-dental images with Convolutional Neural Network (CNN) algorithm, and they also predicted caries along with its two types proximal and occlusal caries, showing 85.6% and 83.6% accurate results, respectively.

Zanella-Calzada et al. [30] discussed deep Artificial Neural Network (ANN) by classifying subjects with the absence of caries to those with caries according to their demographic and dietary factor or nutritional feature (energy, nutrients, and food elements) and predicted accurate results for dental caries with 88% accuracy. Hung et al. [29] used smart phone color photographs, and they used support vector machine (SVM) algorithm on a total of 620 unrestored molar/premolar images. On the 80% training and 20% testing division of dataset, SVM shows 92.37% accuracy. Zanella-Calzada et al. [30] used different types of algorithms of machine learning (SVM, *k*-Nearest Neighbor, Random Forest Regression, and Logistic Regression) on 5,135 dental images. On each algorithm, they divide the dataset into 80% and 20% of training and testing, respectively. Among them, they concluded that SVM shows the highest accuracy, approximately 97.1%. Lee et al. [26] applied Convolutional Neural Networks (CNNs) on a dataset of 2417 images (853 healthy tooth surfaces/1,086 noncavitated carious lesions/431 cavitations/47 automatically excluded images during preprocessing). This study divided the improper division of dataset as they claimed that they divided that dataset into training set (*N* = 1,891/673/870/348) and a test set (*N* = 479/180/216/83). This distribution does not justify any division like 25%, 50%, 75%, and 100% of training as mentioned in the paper. In spite of this, they used CNNs to diagnose correctly with approximately 93.3% accuracy.

Figure 5 presents accuracies of respective studies and success rates of using deep learning with different algorithms in prediction of dental caries and its types (proximal, root caries, and occlusal). Nevertheless, since there are not only three types of dental caries to predict, but there is a variety of types based on tissue involvement, progression type, anatomical site and pathway of caries, further studies should evaluate the diagnosis of other types of caries.

Figure 6 shows the comparison of accuracy according to their algorithms used in the respective study. Devito et al. used Hidden-Layer Perceptron Backpropagation (HLP-BP) and acquired the accuracy of 88.04%. Similarly, Mayank et al., Casalegno et al., Leea et al., Zanella et al., Moutselos et al., Patil et al., Javed et al., and Geetha et al., respectively, used fully convolutional neural network (FCNN), convolutional neural network (CNN), artiﬁcial neural network (ANN), Adaptive Dragonfly algorithm (ADA-NN), Feedforward backpropagation ANN (FFBP-ANN), and backpropagation neural network (BP-NN). Hung et al. and Kühnisch et al. both applied Support Vector Machine (SVM).

Figure 7 indicates that 5 studies out of twelve, those of Mayank et al., Casalegno et al., Leea et al., Kühnisch et al., and Moutselos et al., selected convolutional neural network while 3 out of 12 (Devito et al., Javed et al., and Geetha et al.) went for algorithm backpropagation neural network. One out of 12, Patil et al. selected Adaptive Dragonfly algorithms ADA with combination with neural network. Two out of twelve studies, Hung et al. and Duong et al., used support vector machine. Lastly, Zanella et al. used artificial neural network.

Figure 8(a) represents the distribution of the dataset in the study of Devito et al., in which training size is 80 dental images where the remaining 80 is divided into 40 images for validation and 40 images for testing [19]. Similarly, in (b) section study, Casalegno et al. utilized 185 images as training dataset and 32 as testing data [18]. In section (c), Mayank et al. divide dataset of 3000 images into 2500 as training and 500 as testing. In section (d), Leea et al. also use a dataset of 3000 images, but here they divide the dataset as 2400 images in training dataset and 600 as testing data [27]. In section (e), Zanella et al. divide their dataset of 189 images as 132 images to train and 57 to test the model [31], whereas in (f) study by Moutselos et al., they use a total of 88 images in which they used 79 images to train to the model and 9 images to test that it is itself a small dataset [28]. In section (g), Patil et al. used a very small size of dataset; their results are not reliable due to the usage of small dataset; they use only 45 images, among which 30 images are used for training purpose and 16 images for testing purpose [32]. Figure 8 In (h), Javed et al. use a dataset of 120 images, from which 40 images were used for testing while 80 images were for training [17]. Last, for (i) study, Geetha et al. divide dataset of 105 images as 67 images for training, 17 for validation, and 21 for testing purpose [21].

Figure 9 demonstrates very clearly that for the dental images dataset, backpropagation neural network algorithm is the best-fit choice because from the respective figure neural network algorithm is tested on different datasets and is showing remarkable accuracy compared to the other three algorithms: CNN, ANN, and ADA + NN. Neural network algorithms hits 99% max accuracy while 88.04% min, indicating highest max accuracy and highest min accuracy.

## 5. Conclusion

Based on the results of this systematic review, it is indicated that from twelve studies 9 were found to be providing high level of evidence in the detection between the X-dental images with and without caries. From these studies' result, Neural Network Backpropagation Algorithm is the best-fit choice on dental images dataset that helps in detecting of dental caries with a maximum accuracy of 99%. Considering our findings, further well-designed studies are needed to demonstrate the diagnosis of further types of dental caries that are based on progression (chronic, acute, and arrested), which tells us about severity of caries, virginity of lesion, and extent of caries. AI in the future will emerge as supreme technology to detect other diseases of oral region combinedly and comprehensively because AI will easily analyze big dataset that contain multiple records. All the AI models provide dental professionals reliable information, improving clinical decision making process. Using AI techniques, high-quality-based patient care and innovated research in dentistry can be established.

## Figures and Tables

**Figure 1:** Diagrammatic illustration of Artificial Intelligence Model.

**Figure 2:** PRISMA flow diagram for the systematic review.

**Figure 3:** Size of datasets from year 2008 to year 2022.

**Figure 4:** Data for training and testing in the selected studies.

**Figure 5:** Accuracy chart from 2008 to 2022.

**Figure 6:** Accuracy chart according to their algorithms used in the respective studies.

**Figure 7:** Number of algorithms that are selected by a total 12 studies.

**Figure 8:** Size of datasets used in the selected studies.

**Figure 9:** Maximum and minimum accuracy percentage among twelve algorithms.

**Table 1:** Risk of bias. Red cross indicates no and green tick indicates yes.

Criteria	Author, year											
	Devito et al., 2008	Mayank et al., 2017	Casalegno et al., 2018	Leea et al., 2018	Zanella et al., 2018	Moutselos et al., 2019	Patil et al., 2019	Javed et al., 2019	Hung et al., 2019	Geetha et al., 2020	Duong et al., 2021	Kühnisch et al., 2022
Inclusion criteria	✓	✓	✓	✓		✓			✓	✓	✓	✓
Exclusion criteria	✓	✓	✓	✓	✓		✓	✓	✓	✓	✓	✓
Feature extraction criteria		✓	✓		✓	✓	✓	✓	✓	✓		✓
Description of diagnosis dental caries	✓	✓	✓		✓	✓				✓	✓	✓
Radiographs examination for dental caries diagnosis	✓			✓			✓	✓	✓	✓	✓	✓
Machine learning algorithm description	✓			✓	✓	✓	✓	✓		✓	✓	
Samples of dataset >149	✓	✓	✓	✓	✓			✓	✓		✓	✓
Description of testing and training evaluation					✓							
Statistical and evaluation	✓	✓	✓	✓	✓	✓	✓	✓	✓	✓	✓	✓
Risk of bias	Low	Low	Low	Low	Low	Moderate	Moderate	Moderate	Low	Low	Low	Low

**Table 2:** Characteristic table for the selected studies.

S. no.	Author, year of publication, country	Objective	Algorithm	Language	Dataset size	Accuracy
1	(1) Devito	To diagnose proximal dental caries	Hidden-layer perceptron with backpropagation	English	160 X-dental radiograph	88.4%
	(2) de Souza Barbosa					
	(3) Filho (2008, Brazil)					
2	(1) Mayank	To detect tooth caries in bitewing radiographs	F-CNN	English	3000	70%
	(2) Pratyush Kumar					
	(3) Lalit Pradhan					
	(4) Srikrishna Varadarajan (2017, USA)					
3	(1) Casalegno	To predict occlusal and proximal caries	CNN	English	217 dental images	(1) Occlusal = 83.6%
	(2) Newton					
	(3) Daher					(2) Proximal = 85.6%
	(4) Abdelaziz A. Lodi-Rizzini					
	(5) F. Schürmann					
	(6) I. Krejci					
	(7) H. Markram (2018, Switzerland)					
4	(1) Jae-Hong Leea	To evaluate the efficacy of deep CNN algorithms for detection and diagnosis of dental caries on periapical radiographs	CNN	English	3000 X-dental images	(1) Molar = 89%
	(2) Do-Hyung Kima					
	(3) Seong-Nyum Jeonga				(1) Molar	(2) Premolar = 88%
	(4) Seong-Ho Choib(2018, Korea)				(2) Premolar	
					(3) Both molar and premolar	
						(3) Both molar and premolar = 82%
5	(1) Laura A. Zanella-Calzada	To diagnose caries using socioeconomic and nutritional features as determinants	ANN	English	189 images	69%
	(2) Carlos E. Galván-Tejada					
	(3) Nubia M. Chávez-Lamas					
	(4) Jesús Rivas-Gutierre					
	(5) Rafael Magallanes-Quintanar					
	(6) Jose M. Celaya-Padilla					
	(7) Jorge I. Galván-Tejada					
	(8) Hamurabi Gamboa-Rosales (2018, Mexico)					
6	(1) K. Moutselos	To determine occlusal caries in dental intraoral images	MASK	English	88	(1) MC = most common = 88.9%
	(2) E. Berdouses		(R-CNN)		In-vitro dental images	(2) CPC = center pixel class = 77.8%
	(3) C. Oulis					
	(4) I. Maglogiannis (2019, Greece)					(3) WC = worst class = 66.7%
7	(1) Shashi Kant Patil	To evaluate accurate detection of caries using feature extraction and classification of the dental images along with amalgamation-adaptive dragonfly algorithm (DA) algorithm and neural network (NN) classifier	(1) Adaptive dragonfly algorithm (ADA-NN)	English	120 dental images	Summarizes the performance analysis of proposed ADA-NN classifier over the other conventional classifiers.
	(2) Vaishali Kulkarni					**Test case 1.** Here, the accuracy of the proposed model is 5.55% better than KNN, SVM, NB and LM-NN.
	(3) Archana Bhise (2019, India)		(2) *K*-nearest neighbors (KNN)		40 for each test case	**Test case 2.** ADA model is 11.76% and 52% superior to the existing models like KNN and SVM in terms of accuracy.
						**Test case 3**. The accuracy of the proposed model is 6.30% better than SVM and NB classifier
			(3) Support vector machine (SVM)			
			(4) Naive Bayes (NB)			
			(5) LM-NN			
8	(1) Syed Javed	To predict of post- *Streptococcus mutans* in dental caries	Feedforward backpropagation	English	45 premolar teeth images	99%
	(2) M. Zakirulla		ANN			
	(3) Rahmath Ulla Baig	(as it causes the dental caries)				
	(4) S.M. Asif					
	(5) Allah Baksh Meer (2019, Saudi Arabia)					
9	(1) Man Hung	Application of machine learning for diagnostic prediction of root caries	Support vector machine (SVM)	English	5,135	From all the machine learning algorithms developed, support vector machine (SVM) demonstrated the best performance with an accuracy of 97.1%
	(2) Maren W. Voss					
	(3) Megan N. Rosales		Random forest regression (RF)			
	(4) Wei Li					
	(5) Weicong Su		*k*-nearest neighbors (*k*-NN)			
	(6) Julie Xu					
	(7) Jerry Bounsanga,		Logistic regression			
	(8) Bianca Ruiz-Negrón Evelyn Lauren					
	(9) Frank W. Licari					
	(2019, Jordan)					
10	(1) Geetha K.	To diagnose dental caries	Backpropagation	English	105	97.1%
	(2) S. Aprameya					
	(3) Dharam					
	(4) M. Hinduja (2020, India)					
11	(1) Duc Long Duong	Automated caries detection with smartphone color photography using machine learning	Support vector machine (SVM)	English	620 unrestored molars/premolars	92.37%
	(2) Malitha Humayun Kabir					
	(3) Rong fu Kuo (2021, Taiwan)					
12	(1) J. Kühnisch	Caries detection on intraoral images using artificial intelligence	Convolutional neural networks (CNNs)	English	2,417 peranent teeth	93.3%
	(2) O. Meyer				(1,317 occlusal and 1,100 smooth surfaces)	
	(3) M. Hesenius					
	(4) R. Hickel1					
	(5) V. Gruhn (2022, Germany)					

## Data Availability

No data were used in this study.
